# Can Previous Levels of Physical Activity Affect Risk Factors for Cardiorespiratory Diseases and Functional Capacity after COVID-19 Hospitalization? A Prospective Cohort Study

**DOI:** 10.1155/2022/7854303

**Published:** 2022-04-25

**Authors:** Ariane Aparecida Viana, Alessandro Domingues Heubel, Vanessa Teixeira do Amaral, Stephanie Nogueira Linares, Gustavo Yudi Orikassa de Oliveira, Bruno Martinelli, Audrey Borghi Silva, Renata Gonçalves Mendes, Emmanuel Gomes Ciolac

**Affiliations:** ^1^São Paulo State University (UNESP), School of Sciences, Department of Physical Education, Exercise and Chronic Disease Research Laboratory (ECDR), Bauru, Brazil; ^2^Federal University of São Carlos (UFSCar), Department of Physical Therapy, Cardiopulmonary Physiotherapy Laboratory, São Carlos, Brazil; ^3^Centro Universitário Do Sagrado Coração (UNISAGRADO), Department of Physical Therapy, Bauru, Brazil

## Abstract

**Purpose:**

To evaluate the influence of previous levels of physical activity on hemodynamic, vascular, ventilatory, and functional outcomes after coronavirus disease 2019 (COVID-19) hospitalization.

**Methods:**

Sixty-three individuals with COVID-19 had their clinical status and previous levels (12 month) of physical activity (Baecke Questionnaire of Habitual Physical Activity) assessed at hospital admission. Individuals were then allocated to lower levels of physical activity (ACT_LOWER_; *N* = 22), intermediate levels of physical activity (ACT_INTERMEDIATE_; *N* = 22), or higher levels of physical activity (ACT_HIGHER_; *N* = 19) groups, according to tertiles of physical activity. Resting hemodynamic (heart rate and brachial/central blood pressures) and vascular (carotid-femoral pulse wave velocity, augmentation index, and brachial artery flow-mediated dilation) variables, pulmonary function (spirometry), respiratory muscle strength (maximal respiratory pressures), and functional capacity (handgrip strength, five-time sit-to-stand, timed-up and go, and six-minute walking tests) were measured at 30 to 45 days after hospital discharge.

**Results:**

ACT_LOWER_ showed lower levels (*P* < 0.05) of forced vital capacity, forced expiratory volume in the first second, maximal voluntary ventilation, and maximal expiratory pressure than ACT_HIGHER_. ACT_LOWER_ also had lower (*P* = 0.023) walking distance (~21%,) and lower percentage of predicted walking distance (~20%) at six-minute walking test during follow-up than ACT_INTERMEDIATE_. However, hemodynamic and vascular variables, handgrip strength, five-time sit-to-stand, and timed-up and go were not different among groups.

**Conclusion:**

ACT_LOWER_ showed impaired ventilatory parameters and walking performance when compared with ACT_HIGHER_ and ACT_INTERMEDIATE_, respectively. These results suggest that previous levels of physical activity may impact ventilatory and exercise capacity outcomes 30 to 45 days after COVID-19 hospitalization discharge.

## 1. Introduction

The pandemic of coronavirus disease 2019 (COVID-19) is a public health emergency, with an unprecedented contagious and mortality worldwide [1]. For example, over 28 million cases and over 645 thousand deaths of COVID-19 have been reported in Brazil (as of February 2022) [2]. At the regional level, over 4 million cases and over 192 thousand hospitalizations were confirmed in São Paulo state [2]. In the city of Bauru (São Paulo state, Brazil), there was over 80 thousand confirmed cases, with a mortality rate of 1.7% [2]. Although most cases of COVID-19 are mild, nearly 20% of patients requires hospitalization due to severe manifestations of viral pneumonia, such as dyspnea and respiratory failure [3]. COVID-19 can also cause several extrapulmonary manifestations [4], including injuries in the liver, kidney, heart, vessels, and other organs, mainly in hospitalized patients [5]. The multiorgan injuries and the immobility/isolation during hospitalization can negatively influence posthospitalization recovery period, resulting in reduction of physical fitness, which may negatively impact the functional capacity [6]. In addition, administration of myotoxic medications can promote deconditioning and muscle atrophy [7]. Indeed, skeletal muscle tissues exhibit robust expression of angiotensin-2 converting enzyme [8]. Consequently, skeletal muscle weakness, fatigue, and pain are common symptoms of COVID-19 [9, 10].

Not surprisingly, a multitude of symptoms and abnormalities may persist for several weeks or months after the resolution of COVID-19 acute phase [11]. Previous studies have reported several sequelae and/or persistent symptoms after hospital discharge, such as respiratory (including serious ones as pulmonary fibrosis) and cardiovascular (chest pain, myocarditis, Postural Orthostatic Tachycardia Syndrome…) disorders, physical deconditioning, fatigue, dyspnea, polyneuropathy and myopathy, dysphagia, arthralgia, cognitive disturbances, and decline in quality of life [11, 12]. Studies assessing factors that may influence and/or reduce long-term consequences of severe acute respiratory syndrome coronavirus 2 (SARS-CoV-2) infection are thus welcome.

Regular practice of physical activity (any bodily movement produced by skeletal muscles that results in energy expenditure) is robustly documented as a preventive and therapeutic strategy for several chronic diseases, including those associated with severe COVID-19 and its outcomes [13, 14]. Additionally, regular physical activity improves several parameters of immune function [15, 16]. In this context, high levels of physical activity have been associated with a lower risk of severe COVID-19 outcomes and mortality [17–20]. Indeed, physical activity and functional capacity are associated with lower complications and better recovery to several clinical conditions [21, 22]. Thus, it is reasonable to speculate that previous levels of physical activity may affect COVID-19 sequelae and persistent symptoms.

It is important to note that post-COVID-19 sequelae will potentially dominate medical practice for years [23]. Rehabilitation recommendations for pulmonary, cardiac, musculoskeletal, neurological, and psychological sequelae should be at the forefront of guiding care for the affected population [23]. In middle-aged and older adults, mild to moderate COVID-19 was significantly associated with worsening of mobility and impairments in physical functioning outcomes, even in the absence of hospitalization [24]. A possible reason for these is that the integration and health of pulmonary, cardiovascular, and musculoskeletal systems dictate individual's functional capacity [25], and the multisystemic characteristics of COVID-19 thus affect it negatively.

However, according to our knowledge, little is known about the influence of previous levels of physical activity in functional capacity and health status after COVID-19 hospitalization. This knowledge is important for a better understanding of the effects of COVID-19 on cardiovascular, respiratory, and musculoskeletal systems, as well as for predicting physical and functional prognostic after hospitalization discharge. Thus, the present prospective cohort study was aimed at evaluating the possible influence of previous levels of physical activity on hemodynamic, ventilatory, and functional outcomes after COVID-19 hospitalization discharge.

## 2. Methods

### 2.1. Population and Study Design

This is a prospective, single-center, cohort study, nested whiting a clinical trial (Brazilian Register of Clinical Trials identifier: RBR-9y32yy) testing the acute and chronic cardiorespiratory and functional capacity changes in individuals who were hospitalized due to COVID-19. All participants were assessed in a hospital ward setting (clinical status, coexisting chronic diseases, demographic characteristics, self-reported body weight and height, ethnicity, hemodynamic, and physical activity status), within 72 hours of admission and at 30 to 45 days after hospital discharge (clinical status, hemodynamic and vascular variables, pulmonary function, respiratory muscle strength, and functional capacity). Clinical outcomes during hospitalization were also assessed through medical record.

Inclusion criteria included the following: (1) laboratory-confirmed COVID-19 diagnosis, with SARS-CoV-2 detected by reverse transcriptase-polymerase chain reaction (RT-PCR) test; (2) stable hemodynamics with no use of vasoactive drugs at hospital admission; and (3) Glasgow Coma Scale score of 15 and breathing spontaneously at hospital admission. Pregnant or lactating women, as well as participants with pacemakers, or who have absolute contraindications for physical activity/exercise (i.e., acute myocardial infarction, unstable angina, uncontrolled cardiac arrhythmias, symptomatic severe aortic stenosis, uncontrolled symptomatic heart failure, acute pulmonary embolism/pulmonary infarction, acute myocarditis/pericarditis, or acute aortic dissection) at follow-up evaluation were not included. One-hundred and twenty-one consecutive individuals hospitalized due to suspected COVID-19 at the Hospital State of Bauru (São Paulo state, Brazil), from July 2020 to February 2021, accepted to participate in the study. Thirteen individuals were not included due to negative RT-PCR test. Three individuals were also not included for not matching inclusion criteria at follow-up analysis, and 42 individuals were lost to follow-up due to different reasons. Thus, 63 individuals underwent baseline and follow-up assessments and were included in final analysis. Participants were then allocated to lower levels of physical activity (ACT_LOWER_; *N* = 22), intermediate levels of physical activity (ACT_INTERMEDIATE_; *N* = 22), or higher levels of physical activity (ACT_HIGHER_; *N* = 19) groups, according to tertiles of physical activity measured at hospital admission. The assessed variables were compared among groups (Figure 1). Study procedures were approved by the Research Ethics Committee at School of Sciences of São Paulo State University (CAAE: 32134720.4.1001.5398). All participants received a detailed description of the study and provided their written informed consent before enrollment in the study.

### 2.2. Clinical Assessment

Baseline assessments included a bedside clinical anamnesis and physical examination (within 72 hours of hospital admission) to obtain demographic characteristics, detailed history of disease with time since first symptoms, comorbidities, and use of oxygen therapy. Follow-up clinical assessment included an ambulatory (30 to 45 days after hospital discharge) anamnesis to obtain persistent symptoms and body weight and height measurements (Ramuza™ anthropometric scale; *Ramuza Indústria e Comércio de Balanças Ltda*., Santana do Parnaíba-SP, Brazil). Body mass index (BMI) was calculated as weight/height^2^ (kg/m^2^), and patients were classified into normal weight (BMI 18.5–24.9 kg/m^2^), overweight (BMI 25.0–29.9 kg/m^2^), and obesity (BMI ≥ 30.0 kg/m^2^) [26]. Current smokers were defined as patients who were smoking at the time of study or had stopped smoking during the last month prior to the study. Vital signs such as body temperature (Medior infrared thermometer model MD-33520, Zhejiang Mondial Electronic Technology Co., Ltd., Taizhou, Zhejiang, China), respiratory rate, blood pressure (Omron HEM 7200™, Omron Healthcare Inc., Dalian, China), heart rate (Polar™ H10 heart rate sensor; Polar Electro Inc, Kempele, Finland), and pulse oxygen saturation (SpO2) (G-Tech™ Led finger oximeter; *Accumed Produtos Médico Hospitalares Ltda.*, Duque de Caxias-RJ, Brazil) were assessed at rest, both at baseline and during follow-up.

### 2.3. Levels of Physical Activity

Levels of physical activity were assessed at baseline, during clinical anamnesis, by Baecke Questionnaire of Habitual Physical Activity previously validated to the Brazilian population [27]. Briefly, the questionnaire assessed levels of physical activity in the past 12 months through three dimensions: occupational (8 questions), sport and physical exercises in leisure (4 questions), and leisure-time (4 questions) physical activity. Scores in each dimension range on a five-point Likert scale (from never to always), generating scores from 1 to 5, where higher scores indicate a higher physical activity level. A total activity index was obtained by summing all scores (maximum score = 15), which was used to allocate participants in the three groups.

### 2.4. Arterial Stiffness and Central Pressure

Arterial stiffness and central pressure were assessed during follow-up, after clinical assessment, using a noninvasive automatic device (Complior Analyse™ PWV and Central Pressure Analysis ™; Alam Medical, Saint-Quentin-Fallavier, France), as previously described [28]. Briefly, with the participants at rest in supine position, common carotid and femoral arteries pressure waveforms were recorded noninvasively using a pressure-sensitive transducer. The distance between the recording sites (*D*) was measured in a straight line with a flexible meter and inserted in the equipment's software before waveforms measurements. Carotid-femoral pulse-wave velocity (PWV, calculated as PWV = *D*/*t*, where (*t*) means pulse transit time), augmentation index (AIx, ratio of augmentation pressure expressed as the difference between the second and first pressure peaks in the pulse wave), and central pressure (assessed directly from the carotid pressure waveform, using mean and diastolic pressures to calibrate the carotid signal) were automatically calculated. Pressure waveforms were measured during 10 to 15 cardiac cycles, and the mean was used for the final analysis. All measurements were performed by an experienced observer that was blinded to participants' group assignment.

### 2.5. Endothelial Function

The endothelium-dependent function was assessed, after arterial stiffness/central pressure assessment, using the noninvasive and standardized method of flow-mediated dilation (FMD) [29]. An ultrasound device (SonoSite M-Turbo™; Fujifilm Inc., Bothell, Washington, USA) was used to evaluate blood flow velocity and brachial artery diameter, which were recorded continuously for 1 minute precuff inflation and 3 minutes postcuff release during hyperemia. All assessments were performed by an experienced operator (blinded to participants' group assignment) with more than 100 scans/year, which is suggested to maintain competency with the FMD method [30]. The recommendations for individuals' preparation, technique execution and data acquisition were respected [30]. Doppler blood flow and artery diameter analyses in B-mode video images were performed using an edge-detection and wall tracking software (Brachial Analyzer for Research, Medical Imaging Applications, Coralville, Iowa, USA). The endothelial function was determined by the following formula: FMD (%) = (peak diameter–baseline diameter)/baseline diameter × 100 [31].

### 2.6. Pulmonary Function Testing and Respiratory Muscle Strength

The pulmonary function testing (spirometry) was performed without bronchodilator and using a calibrated and validated portable spirometer (SpiroPro®, Jaeger, Höchberg, Germany), as previously described [28]. Forced vital capacity, forced expiratory volume in one second (FEV_1_), and peak expiratory flow were obtained by asking to the individual an inspiration until total lung capacity and a quick and intense expiration for at least 6 seconds. At least three trials were performed, and the largest values of forced vital capacity and FEV_1_ were determined. All maneuvers were checked for acceptability and reproducibility criteria [32]. Absolute forced vital capacity and FEV_1_ were adjusted to predicted values according to the Brazilian Guidelines for Pulmonary Function Testing [33]. Maximal voluntary ventilation was calculated indirectly using the formula: 37.5 × FEV_1_ + 15.8 [33].

Respiratory muscle strength was measured by analog manovacuometer (Commercial Médica™, São Paulo-SP, Brazil). The maximal inspiratory pressure was measured with scale of ±120 cm H_2_O, from residual volume up to the total lung capacity. The maximal expiratory pressure was measured from the total lung capacity, with the patient being instructed to fully inhale and exhale with maximum effort. At least three consecutive trials were carried out, with an interval of one minute between them. The value considered was the highest among the three measurements (except if it was the last) [34]. These variables were measured during follow-up, after pulmonary function testing, with participants at seated position.

### 2.7. Functional Capacity–Different Aspects of Functional Capabilities

Functional capacity was assessed through muscle strength (handgrip strength), functional tests [five-time sit-to-stand (FTSTS) and timed-up and go (TUG)], and walking performance [six-minute walking test (6MWT)], as previously described [28] and briefly detailed below.

*Handgrip strength*: handgrip strength was measured during follow-up (after pulmonary function assessment), using a hydraulic dynamometer (Jamar™; Bolingbrook, Illinois, USA). To perform the measurement, the patient was at seated position, with the elbow flexed at 90 degrees and wrist in neutral. Three measures were performed for each hand, and the greater of the two averaged values was recorded as the final grip strength value [35].

*FTSTS*: lower limb muscle strength/power was measured during follow-up, after handgrip strength assessment, by the FTSTS test, as previously described [36].

*TUG*: balance/agility was measured during follow-up, after FTSTS test, by the TUG test, as previously described [36].

*6MWT*: the 6MWT was performed during follow-up, after TUG test, on a 30 m length flat surface, using cones and measure tape to mark the ground [37], and following the recommendations of the European Respiratory Society/American Thoracic Society [38]. Blood pressure (Omron HEM 7200™, Omron Healthcare Inc., Dalian, China) was measured before, immediately after, and after 2 min of recovery. Heart rate (Polar™ H10 heart rate sensor; Polar Electro Inc, Kempele, Finland) and SpO_2_ (G-Tech™ Led finger oximeter; *Accumed Produtos Médico Hospitalares Ltda.*, Duque de Caxias-RJ, Brazil) were measured before, every 2 min of exercise (2, 4, and 6 min), and at 1 min of recovery. The average of heart rate and SpO_2_ measured every 2 min of exercise was considered exercise heart rate and exercise SpO_2_, respectively. Absolute (total distance walked during test) and relative (percentage of predicted distance) [39] values were used to assess walking performance. The prevalence of partial oxygen desaturation during the exercise phase was measured as a reduction ≤4% in SpO_2_ during any moment of walking when compared to preexercise levels.

### 2.8. Statistical Analysis

Data are reported as mean (95% confidence interval). Data normality and homoscedasticity were tested using Shapiro-Wilk and Leveneʼs tests, respectively. Chi-square was used to indicate difference among groups in categorical variables. One-way ANOVA and Kruskal Wallis were used to indicate differences among groups in normally distributed and nonnormally distributed variables, respectively. The Bonferroni and Dunn's *post hoc* analyses were used to identify significant differences indicated by one-way ANOVA and Kruskal Wallis, respectively. Statistical software SPSS 17.0™ (SPSS Inc., Chicago, IL, USA) was used to perform the statistical analyses. The level of significance was set at *P* < 0.05.

## 3. Results

The clinical characteristics and detailed description of the groups at baseline are presented in Table 1. Total, occupational, sport, and leisure levels of physical activity were significantly different among groups (*P* < 0.001). There was no significant difference among the groups for almost all other variables at baseline. Exception for age and hypertension prevalence, with the ACT_HIGHER_ being younger than ACT_LOWER_ (~11 years, *P* = 0.01), and with lower prevalence of hypertension in ACT_HIGHER_ (26%) than both ACT_LOWER_ (64%) and ACT_INTERMEDIATE_ (55%).

During follow-up, 83% of the participants had at least one persistent symptom of COVID-19, with no significant difference among the groups (Table 2). The six most frequent COVID-19-related persistent symptoms were fatigue (68%), dyspnea (40%), cough (25%), myalgia (22%), headache (19%), and chest pain (16%). Resting cardiovascular (brachial and central blood pressure and heart rate and arterial stiffness) and respiratory parameters (respiratory rate and SpO_2_) were not different among groups and were within normal ranges. FMD was also not different among groups. Absolute levels of forced vital capacity, FEV_1_, and maximal voluntary ventilation were lower (*P* < 0.05) in the ACT_LOWER_ than in the ACT_HIGHER_ (forced vital capacity: ~23%, *P* = 0.022; FEV_1_: ~24%, *P* = 0.017; maximal voluntary ventilation: ~21%, *P* = 0.017). However, relative levels (% of predicted) of forced vital capacity and FEV_1_ were not different among the groups. Absolute levels of maximal inspiratory pressure were lower in the ACT_LOWER_ than in the ACT_HIGHER_ (~31%, *P* = 0.035), and absolute levels of maximal expiratory pressure were lower in the ACT_LOWER_ than in the ACT_HIGHER_ (~34%, *P* = 0.017) and tended to be lower in the ACT_INTERMEDIATE_ than in the ACT_HIGHER_ (~26%, *P* = 0.074). However, only relative levels (% of predicted) of maximal expiratory pressure were significant different among the groups, where lower levels were found in the ACT_LOWER_ than in the ACT_HIGHER_ (~26%, *P* = 0.044).

Performance and physiological response to 6MWT were also different among groups during follow-up. ACT_LOWER_ had lower walking distance (~21%, *P* = 0.023) and lower percentage of predicted walking distance (~20%, *P* = 0.023) than ACT_INTERMEDIATE_ (Figures 2(a) and 2(b)). Preexercise heart rate, blood pressure, and SpO_2_, as well as blood pressure response during exercise and recovery were not significantly different among groups (Figures 2(c)–2(e)). However, it was found a tendency toward lower heart rate during exercise (~17 bpm, *P* = 0.06) and recovery (~11 bpm, *P* = 0.062) in the ACT_LOWER_ than in the ACT_INTERMEDIATE_ (Figure 2(c)), as well as a tendency toward lower exercise SpO_2_ (~4%, *P* = 0.075) in the ACT_LOWER_ than in the ACT_HIGHER_ (Figure 2(e)). Although the ACT_LOWER_ showed lower walking distance (~16%), percentage of predicted walking distance (~12%), exercise heart rate (~13 bpm), and recover heart rate (~8 bpm) than the ACT_HIGHER_, these differences were not statistically different. The same occurred with the exercise SpO_2_, where the lower levels (~3%) observed in the ACT_LOWER_ than in the ACT_INTERMEDIATE_ were not statistically different. The prevalence of partial oxygen desaturation during the exercise phase of 6MWT was higher in the ACT_LOWER_ (41%), followed by the ACT_INTERMEDIATE_ (32%) and ACT_HIGHER_ (16%), respectively. However, these differences were not statistically different (*P* = 0.211). There were no significant differences among groups in handgrip strength, TUG, and FTSTS during follow-up (Figure 3).

## 4. Discussion

COVID-19 results in a broad array of pulmonary and extrapulmonary clinical manifestations with functional capacity impairment (e.g., mobility decline, reduced exercise tolerance, lung damage, circulatory limitation, muscle weakness, and myopathy) [40–42]. Previous studies have shown that high levels of physical activity are associated with a lower risk of acute severe COVID-19 outcomes (i.e., hospitalization, ICU admission, IMV, cardiovascular events…) and mortality [16–20]. However, to our knowledge, this is the first prospective cohort study assessing the role of previous levels of physical activity on cardiovascular, ventilatory, and functional outcomes after COVID-19 hospitalization discharge.

The present study showed that absolute levels of forced vital capacity, FEV_1_, maximal voluntary ventilation and maximal inspiratory pressure, as well as absolute and relative levels of maximal expiratory pressure were lower in the ACT_LOWER_ than in the ACT_HIGHER_. In addition, ACT_LOWER_ also showed lower 6MWT distance and percentage of predicted 6MWT distance than ACT_INTERMEDIATE_. Indeed, a tendency toward lower exercise and recovery heart rate in the ACT_LOWER_ than in the ACT_INTERMEDIATE_, as well as a tendency toward lower exercise SpO_2_ in the ACT_LOWER_ than in the ACT_HIGHER_ were also found during follow-up. On the other hand, resting respiratory, hemodynamic, vascular, and functional (FTSTS and TUG) parameters were not different among the groups during follow-up.

The participants' respiratory variables at rest were not different among the groups and were whiting normal clinical parameters during follow-up (Table 2). Compared with baseline, all groups increased SpO_2_ (~3.5%) and decreased respiratory rate (~5.6 bpm). Resting hemodynamic and vascular variables were also within normal limits and were not different among the groups, suggesting that the previous levels of physical activity did not affect resting respiratory, hemodynamic, and vascular parameters 30 to 45 after hospital discharge. However, although the parameters were not significantly different among the groups, ACT_HIGHER_ presented lower levels of brachial and central blood pressures, and pulse-wave velocity (Table 2), which is probably due to the lower prevalence of hypertension in this group.

Previous longitudinal study showed that increases in systemic inflammation are associated with declines in lung function [43]. Individuals with severe COVID-19 have presented a cytokine storm [44], independently if admitted or not admitted to the intensive care unit during hospitalization. The inflammatory response and accumulation of proinflammatory cytokines may contribute to muscle wasting by stimulating protein catabolism, affecting respiratory muscles, and potentially contributing to impaired pulmonary function [45]. Thus, a reduction in respiratory variables may be expected in individuals hospitalized due to COVID-19 and may be referred as symptoms of fatigue and weakness in the postacute phase. These are the most prevalent persistent symptoms with 64% to 68% of prevalence [46–48], which is in line with the 68% of fatigue prevalence we found during follow-up, which were not significantly different among the groups.

We found normal levels of FEV_1_/FVC ratio (>80%) in all groups during follow-up. However, there were significant differences between ACT_LOWER_ and ACT_HIGHER_ in several spirometry parameters. Absolute levels of FEV_1_ (~24%), forced vital capacity (~23%), and maximal voluntary ventilation (~21%) were lower in the ACT_LOWER_ than in the ACT_HIGHER_. FEV_1_ and forced vital capacity are parameters associated with restrictive ventilatory disorders that may be caused by several factors such as alterations in lung parenchyma, pleura, chest wall, or neuromuscular apparatus [49]. In our study, patients in the ACT_LOWER_ and ACT_HIGHER_ did not require mechanical ventilation during hospitalization. According to a recent study, patients with moderate or severe COVID-19 mainly developed mild-to-severe pulmonary fibrosis, and the severe lung inflammation (IL-6 levels in the acute stage) has been associated with more extensive and severe residual pulmonary fibrosis [50]. A good finding was that chest high-resolution computed tomography showed that the affected area was significantly improved 30 days after discharge compared with at discharge [50]. We did not assess IL-6 levels at the acute stage or chest high-resolution computed tomography at the follow-up. Furthermore, the age difference between the ACT_LOWER_ and ACT_HIGHER_ may be a confounding factor.

On the other hand, a study assessing the association of physical activity with pulmonary function in adults found that physically active individuals showed higher levels of forced vital capacity and FEV_1_ than physically inactive individuals [51]. Endurance-trained individuals had greater maximal voluntary ventilation, which is an adaptation to maintain a greater and prolonged ventilation for meeting the gas exchange demands of exercise [52]. Thus, it is possible that the present lower spirometry parameters in the ACT_LOWER_ than in the ACT_HIGHER_ is a consequence of the previous levels of physical activity, suggesting that lower previous levels of physical activity can make the patients more susceptible to complications after COVID-19 hospitalization discharge.

Previous study assessing 379 patients after 4 months of COVID-19 hospitalization found a decreased respiratory muscle strength, with the participants showing relative maximal inspiratory and expiratory pressures at 58% and 79% of predicted levels, respectively [53]. ,Our findings also showed decreased respiratory muscle strength in all groups (relative maximal inspiratory and expiratory pressures below 80% of predicted levels). The possible reasons for these decreased respiratory muscle strength after hospital discharge include (a) deconditioning as a result of immobility during hospital stay; (b) indirect damage to musculoskeletal tissue, including respiratory muscles [54]; (c) direct damage to diaphragmatic myofibers as a result of viral invasion via angiotensin-2 converting enzyme [55]; and (d) limited physical activity secondary to social distancing and lockdown [56]. However, it is important to note that the relative maximum expiratory pressure was ~26% lower in the ACT_LOWER_ than in the ACT_HIGHER_ in the present study, suggesting that a previous higher level of physical activity may be a better predictor of respiratory muscle strength, despite of the above-mentioned interferences.

Although there are several gaps regarding the knowledge about exercise capacity and health status post-COVID-19 hospitalization, several studies have suggested an important impact of physical activity levels and COVID-19 disease outcomes [17–20]. In addition, the previous experience with SARS, a severe viral respiratory syndrome similar to COVID-19, showed that patients who contracted this pathology had variables degrees of cardiorespiratory, quality of life, and muscle performance abnormalities after 1-year of follow-up. Indeed, 23.7% showed a reduction in exercise capacity even one year after hospital discharge, when compared to the predicted levels for healthy individuals at same age [57]. In the present study, we found lower levels of 6MWT distance (~21%) and percentage of predicted 6MWT distance (~20%) in the ACT_LOWER_ than in the ACT_INTERMEDIATE_ during follow-up. Indeed, the lower levels of 6MWT distance (~16%) and percentage of predicted 6MWT distance (~12%) in the ACT_LOWER_ than in the ACT_HIGHER_ deserve attention, despite of the absence of statistically significance. Interestingly, higher muscle strength and respiratory function did not result in significant 6MWT distance in the ACT_HIGHER_. One possible explanation may be the multisystemic characteristic of COVID-19. The performance of functional tests requires the integration of multiple physiologic systems and may not be affected only by the respiratory system. The combined effect of detraining and COVID-19 sequelae may influence the capacity to perform exercise [58], and both respiratory and leg muscles are vulnerable to a wide range of systemic disorders that can lead to impaired strength and mobility [59]. Another important point to be considered is our small sample size.

It is also important to note that we found a tendency toward lower exercise and recovery heart rate in the ACT_LOWER_ than in the ACT_INTERMEDIATE_, as well as a tendency toward lower exercise SpO_2_ in the ACT_LOWER_ than in the ACT_HIGHER_ during follow-up. Interestingly, the prevalence of partial oxygen desaturation during the exercise phase of 6MWT was not statistically different among the groups (*P* = 0.211), it was also higher in ACT_LOWER_ (41%) than both ACT_INTERMEDIATE_ (32%) and ACT_HIGHER_ (16%). These findings suggest that the previous lower levels of physical activity may result in worse exercise capacity during COVID-19 recovery and consequently make the patient more susceptible to complications.

Previous study with survivors from COVID-19 pneumonia showed that reduced oxygen content and extraction secondary to anemia and myopathic changes, rather than respiratory, pulmonary, vascular, or cardiac impairments, were the main contributors to reduced exercise capacity on the day before hospital discharge [7]. In line with the role of peripheral factors on exercise capacity, fatigue or muscle weakness was the most common persistent symptoms (63%) after 6 months COVID-19 onset [60]. In this context, it is possible that a suboptimal oxygen extraction may be associated with the lower 6MWT walking distance and percentage of predicted distance found in the ACT_LOWER_. It has been suggested that the combined effect of detraining and COVID-19 symptoms may influence the arousal of postviral fatigue syndrome, thus influencing the capacities to perform exercise [58]. According to the present findings, the previous level of physical activity is also an important factor affecting exercise capacity 30 to 45 days after COVID-19 hospitalization discharge. Therefore, it is reasonable to suggest that the practice of physical activity should be intensified during COVID-19 pandemic, for both general population and individuals recovering from COVID-19, as a measure of reducing the risk of pulmonary and exercise capacity abnormalities.

Finally, our study has some limitations. First, the small sample size in each group does not warrant similar results in other COVID-19 populations, mainly those with higher prevalence of comorbidities. Second, we assessed individuals that were hospitalized in a single hospital and that were in the first infection and not vaccinated. In addition, until the end of data collection, there was no record of circulation of viral variants in the participating hospital. These factors may limit extrapolations to other healthcare settings, patients that are vaccinated or at second infection, as well as infected for recent variants. Third, we also did not assess biomarkers at the follow-up, which can be used to quantify immunologic dysfunction and cardiovascular risk. Therefore, we were unable to determine whether exercise capacity was impaired only due to abnormalities in cardiorespiratory and muscle performance, or also by a dysregulation in inflammatory or immune responses.

## 5. Conclusions

ACT_LOWER_ showed impaired ventilatory and walking performance 30 to 45 days after hospital discharge due to COVID-19 hospitalization, when compared with ACT_HIGHER_ and ACT_INTERMEDIATE_, respectively. However, resting respiratory, hemodynamic, vascular, and functional (FTSTS and TUG) parameters were not different among the groups during follow-up. Future studies assessing the long-term impact of previous levels of physical activity on ventilatory and exercise capacity outcomes, as well as its clinical consequences, are welcome.

## Figures and Tables

**Figure 1:** Flowchart of the study recruitment. RT-PCR: Reverse transcriptase-polymerase chain reaction; ACT_LOWER_: Lower levels of physical activity group; ACT_INTERMEDIATE_: Intermediate levels of physical activity group; ACT_HIGHER_: Higher levels of physical activity group.

**Figure 2:** Six-minute walking test distance (a), percentage of predicted distance (b), heart rate (c), blood pressure (d), and pulse oxygen saturation (e) during follow-up. ACT_LOWER_: Lower levels of physical activity group; ACT_INTERMEDIATE_: Intermediate levels of physical activity group. ACT_HIGHER_: Higher levels of physical activity group. Asterisk denotes significant difference from the lower physical activity group (^∗^*P* < 0.05). Circle denotes tendency toward difference between lower and intermediate (°*P* = 0.06) or high (•*P* = 0.075) physical activity groups.

**Figure 3:** Functional parameters during follow-up. ACT_LOWER_: Lower levels of physical activity group; ACT_INTERMEDIATE_: Intermediate levels of physical activity group; ACT_HIGHER_: Higher levels of physical activity group.

**Table 1:** Participants' characteristics at baseline.

Variables	Physical activity groups (tertile)			*P*
	Lower (*N* = 22)	Intermediate (*N* = 22)	Higher (*N* = 19)	
Age (yr)	58 (53–62)	52 (47–57)	47 (41–53)^∗^	0.013
Gender (male/female)	8/14	10/12	10/9	0.575
Race (*N*, white/black/mixed/indigenous)	17/4/0/1	17/3/1/1	11/4/4/0	0.233
BMI (kg/m^2^)	34.3 (30.9–37.7)	32.8 (30.2–35.4)	32.4 (28.8–35.9)	0.638
Tabagism (*N*, never/current/former)	7/1/4	16/2/4	15/2/2	0.900
Comorbidities [*N* (%)]	16 (73)	15 (68)	10 (53)	0.376
CVD [*N* (%)]	5 (23)	5 (23)	1 (5)	0.099
DM [*N* (%)]	6 (27)	4 (18)	1 (5)	0.179
Dyslipidemia [*N* (%)]	2 (9)	2 (9)	1 (5)	0.875
Hypertension [*N* (%)]	14 (64)	12 (55)	5 (26)	0.048
Hypothyroidism [*N* (%)]	4 (19)	2 (9)	0 (0)	0.141
Obesity [*N* (%)]	16 (73)	14 (64)	13 (68)	0.811
Respiratory disease [*N* (%)]	4 (18)	2 (9)	2 (11)	0.626
Other diseases [*N* (%)]	5 (23)	5 (23)	2 (11)	0.527
Hospital stays (days)	7.8 (5.7–9.9)	7.9 (5.2–10.7)	5.3 (4.1–6.4)	0.083
Adverse events [*N* (%)]	5 (23)	2 (9)	1 (5)	0.202
ICU admission [*N* (%)]	4 (18)	2 (9)	1 (5)	0.394
IMV [*N* (%)]	0 (0)	2 (9)	0 (0)	0.146
Cardiovascular events [*N* (%)]	2 (9)	0 (0)	0 (0)	0.146
Non-cardiovascular events [*N* (%)]	1 (5)	1 (5)	0 (0)	0.640
Physical activity levels				
Total	5.8 (5.5–6.1)	7.2 (7.1–7.5)^∗∗^	8.9 (8.6–9.3)^†^	< 0.001
Occupational	2.4 (2.1–2.8)	2.8 (2.6–3.1)^∗∗^	3.4 (3.0–3.7)^†^	0.001
Sport	1.9 (1.7–2.1)	2.3 (2.0–2.7)^∗∗^	2.7 (2.5–3.0)^†^	< 0.001
Leisure	1.6 (1.5–1.8)	2.1 (1.9–2.3)^∗∗^	3.1 (2.8–3.4)^†^	< 0.001

Ordinal data are presented as mean (95% confidence interval). BMI: Body mass index; CVD: Cardiovascular disease; DM: Diabetes mellitus; ICU: Intensive care unit; IMV: Invasive mechanical ventilation. Asterisk denotes significant difference from lower physical activity group (^∗^*P* = 0.01;  ^∗∗^*P* < 0.001); dagger denotes significant difference from lower and intermediate physical activity groups (*P* < 0.001).

**Table 2:** Clinical, hemodynamic and respiratory variables during follow-up.

Variables	Physical activity groups (tertile)			*P*
	Lower (*N* = 22)	Intermediate (*N* = 22)	Higher (*N* = 19)	
Days after hospital discharge	38 (34–41)	37 (33–40)	35 (33–38)	0.608
Persistent symptoms [*N* (%)]	18 (82)	18 (82)	16 (84)	0.974
Heart rate (bpm)	76 (70–81)	85 (78–92)	79 (71–86)	0.110
SpO_2_ (%)	96 (95–97)	97 (96–97)	96 (96–97)	0.444
Respiratory rate (bpm)	17 (15–19)	17 (15–19)	15 (13–17)	0.131
Brachial blood pressure				
Systolic (mmHg)	135 (124–146)	129 (122–137)	122 (115–129)	0.114
Diastolic (mmHg)	80 (74–87)	84 (79–89)	76 (71–81)	0.145
Central blood pressure				
Systolic (mmHg)	129 (116–141)	122 (111–133)	114 (107–120)	0.146
Diastolic (mmHg)	80 (73–86)	83 (78–88)	77 (72–82)	0.275
Arterial stiffness				
Pulse-wave velocity (m/s)	9.2 (8.0–10.4)	8.5 (7.8–9.2)	7.8 (6.8–9.0)	0.167
Aix	15.2 (8.1–22.3)	12.9 (5.0–20.1)	13.6 (5.2–22.0)	0.903
Vascular measures				
FMD (mm)	0.25 (0.21–0.28)	0.26 (0.23–0.30)	0.29 (0.21–0.36)	0.509
FMD relative (%)	5.69 (4.68–6.70)	6.43 (5.35–7.50)	6.55 (5.02–8.08)	0.515
Pulmonary function				
Forced vital capacity (l)	3.11 (2.68–3.54)	3.52 (3.13–3.91)	4.08 (3.38–4.78)^∗^	0.026
Forced vital capacity relative (% predicted)	91 (83–99)	99 (91–107)	103 (91–114)	0.158
FEV_1_ (l)	2.56 (2.24–2.89)	2.95 (2.66–3.23)	3.37 (2.76–3.98)^∗^	0.021
FEV_1_ relative (% predicted)	95 (86–104)	103 (94–111)	103 (91–116)	0.403
FEV_1_/forced vital capacity (l)	84 (79–88)	84 (82–87)	82 (78–86)	0.641
Maximal voluntary ventilation (l)	112 (100–124)	126 (115–137)	142 (119–165)^∗^	0.022
Peak expiratory flow (l/s)	5.27 (4.19–6.36)	7.13 (5.83–8.43)	7.07 (5.47–8.67)	0.066
Maximal inspiratory pressure (cmH_2_O)	53 (41–65)	69 (57–80)	77 (60–94)^∗^	0.034
Maximal inspiratory pressure relative (% predicted)	54 (43–65)	67 (59–75)	70 (56–85)	0.094
Maximal expiratory pressure (cmH_2_O)	53 (40–67)	59 (46–71)	80 (66–94)^∗^°	0.015
Maximal expiratory pressure relative (% predicted)	54 (43–66)	57 (48–66)	73 (61–84)^∗^	0.032

Ordinal data are presented as mean (95% confidence Interval). FEV_1_: Forced expiratory volume in the first second; SpO_2_: Peripheral oxygen saturation. Asterisk denotes significant difference from lower physical activity group (^∗^*P* < 0.05). Circle denotes tendency toward difference from intermediate physical activity group (°*P* = 0.074).

## Data Availability

The data used to support the findings of this study are available through the corresponding author upon reasonable request.

## Additional Points

*Highlights*. (i) Previous levels of physical activity were not associated with resting heart rate, resting blood pressure (brachial and central), arterial stiffness, endothelial function, handgrip strength, and five-time sit-to-stand and timed-up and go performance. (ii) Individuals in the lowest tertile of physical activity showed impaired forced vital capacity, forced expiratory volume in the first second, and maximal expiratory pressure and walking performance, when compared with individuals in the higher and intermediate tertiles of physical activity. (iii) Previous levels of physical activity appear to impact ventilatory and walking performance outcomes 30 to 45 days after COVID-19 hospitalization discharge

## References

[1] World Health Organization (2021). Coronavirus disease (COVID-19). *Weekly epidemiological update*.

[2] Brazil, Ministry of health Coronavirus Panel. https://covid.saude.gov.br/.

[3] Wu Z., McGoogan J. M. (2020). Characteristics of and important lessons from the coronavirus disease 2019 (COVID-19) outbreak in China: summary of a report of 72 314 cases from the Chinese Center for Disease Control and Prevention. *Journal of the American Medical Association*.

[4] Gupta A., Madhavan M. V., Sehgal K. (2020). Extrapulmonary manifestations of COVID-19. *Nature Medicine*.

[5] Wang X., Fang X., Cai Z. (2020). Comorbid chronic diseases and acute organ injuries are strongly correlated with disease severity and mortality among COVID-19 patients: a systemic review and meta-analysis. *Research*.

[6] Thomas P., Baldwin C., Bissett B. (2020). Physiotherapy management for COVID-19 in the acute hospital setting: clinical practice recommendations. *Journal of Physiotherapy*.

[7] Baratto C., Caravita S., Faini A. (2021). Impact of COVID-19 on exercise pathophysiology: a combined cardiopulmonary and echocardiographic exercise study. *Journal of Applied Physiology*.

[8] Nehme A., Cerutti C., Dhaouadi N. (2015). Atlas of tissue renin-angiotensin-aldosterone system in human: a transcriptomic meta-analysis. *Scientific Reports*.

[9] Jin M., Tong Q. (2020). Rhabdomyolysis as potential late complication associated with COVID-19. *Emerging Infectious Diseases*.

[10] Sun P., Lu X., Xu C., Sun W., Pan B. (2020). Understanding of COVID-19 based on current evidence. *Journal of Medical Virology*.

[11] Nalbandian A., Sehgal K., Gupta A. (2021). Post-acute COVID-19 syndrome. *Nature Medicine*.

[12] Carda S., Invernizzi M., Bavikatte G. (2020). COVID-19 pandemic. What should physical and rehabilitation medicine specialists do? A clinician’s perspective. *European Journal of Physical and Rehabilitation Medicine*.

[13] Grasselli G., Zangrillo A., Zanella A. (2020). Baseline characteristics and outcomes of 1591 patients infected with SARS-CoV-2 admitted to ICUs of the Lombardy Region, Italy. *Journal of the American Medical Association*.

[14] Zhou F., Yu T., Du R. (2020). Clinical course and risk factors for mortality of adult inpatients with COVID-19 in Wuhan, China: a retrospective cohort study. *Lancet*.

[15] Ciolac E. G., Rodrigues da Silva J. M., Vieira R. P. (2020). Physical exercise as an immunomodulator of chronic diseases in aging. *Journal of Physical Activity & Health*.

[16] Burtscher J., Millet G. P., Burtscher M. (2021). Low cardiorespiratory and mitochondrial fitness as risk factors in viral infections: implications for COVID-19. *British Journal of Sports Medicine*.

[17] de Souza F. R., Motta-Santos D., Dos Santos Soares D. (2021). Association of physical activity levels and the prevalence of COVID-19-associated hospitalization. *Journal of Science and Medicine in Sport*.

[18] Sallis R., Young D. R., Tartof S. Y. (2021). Physical inactivity is associated with a higher risk for severe COVID-19 outcomes: a study in 48 440 adult patients. *British Journal of Sports Medicine*.

[19] Tavakol Z., Ghannadi S., Tabesh M. R. (2021). Relationship between physical activity, healthy lifestyle and COVID-19 disease severity; a cross-sectional study. *Journal of Public Health*.

[20] Yates T., Razieh C., Zaccardi F. (2021). Obesity, walking pace and risk of severe COVID-19 and mortality: analysis of UK Biobank. *International Journal of Obesity*.

[21] Schonborn J. L., Anderson H. (2019). Perioperative medicine: a changing model of care. *BJA Education*.

[22] Assouline B., Cools E., Schorer R., Kayser B., Elia N., Licker M. (2021). Preoperative exercise training to prevent postoperative pulmonary complications in adults undergoing major surgery. A systematic review and meta-analysis with trial sequential analysis. *Annals of the American Thoracic Society*.

[23] Barker-Davies R. M., O'Sullivan O., Senaratne K. P. P. (2020). The Stanford Hall consensus statement for post-COVID-19 rehabilitation. *British Journal of Sports Medicine*.

[24] Beauchamp M. K., Joshi D., McMillan J. (2022). Assessment of functional mobility after COVID-19 in adults aged 50 years or older in the Canadian longitudinal study on aging. *JAMA Network Open*.

[25] Arena R., Myers J., Williams M. A. (2007). Assessment of functional capacity in clinical and research settings: a scientific statement from the American Heart Association Committee on exercise, rehabilitation, and prevention of the council on clinical cardiology and the council on cardiovascular nursing. *Circulation*.

[26] World Health Organization (2000). *Obesity: preventing and managing the global epidemic. Report of a WHO consultation*.

[27] Florindo A. A., Latorre M. R. D. O. (2003). Validation and reliability of the Baecke Questionnaire for the evaluation of habitual physical activity in adult men. *Revista Brasileira de Medicina do Esporte*.

[28] do Amaral V. T., Viana A. A., Heubel A. D. (2022). Cardiovascular, respiratory and functional effects of tele-supervised home-based exercise training in individuals recovering from COVID-19 hospitalization: A randomized clinical trial. *medRxiv*.

[29] Thijssen D. H. J., Bruno R. M., van Mil A. C. C. M. (2019). Expert consensus and evidence-based recommendations for the assessment of flow-mediated dilation in humans. *European Heart Journal*.

[30] Corretti M. C., Anderson T. J., Benjamin E. J. (2002). Guidelines for the ultrasound assessment of endothelial-dependent flow- mediated vasodilation of the brachial artery: a report of the International Brachial Artery Reactivity Task Force. *Journal of the American College of Cardiology*.

[31] Harris R. A., Nishiyama S. K., Wray D. W., Richardson R. S. (2010). Ultrasound assessment of flow-mediated dilation. *Hypertension*.

[32] Graham B. L., Steenbruggen I., Miller M. R. (2019). Standardization of spirometry 2019 update. An official American Thoracic Society and European Respiratory Society technical statement. *American Journal of Respiratory and Critical Care Medicine*.

[33] Pereira C. A. C. (2002). Espirometria. *Diretrizes para Testes de Função Pulmonar*.

[34] Neder J. A., Andreoni S., Lerario M. C., Nery L. E. (1999). Reference values for lung function tests: II. Maximal respiratory pressures and voluntary ventilation. *Brazilian Journal of Medical and Biological Research*.

[35] Fess E. E., Casanova J. S. (1992). Grip strength. *Clinical Assessment Recommendations*.

[36] Rodrigues da Silva J. M., de Rezende M. U., Spada T. C. (2017). Educational program promoting regular physical exercise improves functional capacity and daily living physical activity in subjects with knee osteoarthritis. *BMC Musculoskeletal Disorders*.

[37] Negreiros A., Padula R. S., Andrea Bretas Bernardes R., Moraes M. V., Pires R. S., Chiavegato L. D. (2017). Predictive validity analysis of six reference equations for the 6-minute walk test in healthy Brazilian men: a cross-sectional study. *Brazilian Journal of Physical Therapy*.

[38] Singh S. J., Puhan M. A., Andrianopoulos V. (2014). An official systematic review of the European Respiratory Society/American Thoracic Society: measurement properties of field walking tests in chronic respiratory disease. *The European Respiratory Journal*.

[39] Iwama A. M., Andrade G. N., Shima P., Tanni S. E., Godoy I., Dourado V. Z. (2009). The six-minute walk test and body weight-walk distance product in healthy Brazilian subjects. *Brazilian Journal of Medical and Biological Research*.

[40] Bellan M., Soddu D., Balbo P. E. (2021). Respiratory and psychophysical sequelae among patients with COVID-19 four months after hospital discharge. *JAMA Network Open*.

[41] Groff D., Sun A., Ssentongo A. E. (2021). Short-term and long-term rates of postacute sequelae of SARS-CoV-2 infection: a systematic review. *JAMA Network Open*.

[42] Medrinal C., Prieur G., Bonnevie T. (2021). Muscle weakness, functional capacities and recovery for COVID-19 ICU survivors. *BMC Anesthesiology*.

[43] Ahmadi-Abhari S., Kaptoge S., Luben R. N., Wareham N. J., Khaw K. T. (2014). Longitudinal association of C-reactive protein and lung function over 13 years: the EPIC-Norfolk study. *American Journal of Epidemiology*.

[44] Huang C., Wang Y., Li X. (2020). Clinical features of patients infected with 2019 novel coronavirus in Wuhan, China. *Lancet*.

[45] Zhang P., Wu H. M., Shen Q. Y., Liu R. Y., Qi X. M. (2016). Associations of pulmonary function with serum biomarkers and dialysis adequacy in patients undergoing peritoneal dialysis. *Clinical and Experimental Nephrology*.

[46] Cheng D., Calderwood C., Skyllberg E., Ainley A. (2021). Clinical characteristics and outcomes of adult patients admitted with COVID-19 in East London: a retrospective cohort analysis. *BMJ Open Respiratory Research*.

[47] D'Cruz R. F., Waller M. D., Perrin F. (2021). Chest radiography is a poor predictor of respiratory symptoms and functional impairment in survivors of severe COVID-19 pneumonia. *ERJ Open Research*.

[48] Halpin S. J., McIvor C., Whyatt G. (2021). Postdischarge symptoms and rehabilitation needs in survivors of COVID-19 infection: a cross-sectional evaluation. *Journal of Medical Virology*.

[49] National Center for Biotechnology Information-MedGen Restrictive ventilatory defect definition. https://www.ncbi.nlm.nih.gov/medgen/478856.

[50] Zou J. N., Sun L., Wang B. R. (2021). The characteristics and evolution of pulmonary fibrosis in COVID-19 patients as assessed by AI-assisted chest HRCT. *PLoS One*.

[51] Luzak A., Karrasch S., Thorand B. (2017). Association of physical activity with lung function in lung-healthy German adults: results from the KORA FF4 study. *BMC Pulmonary Medicine*.

[52] Hackett D. A. (2020). Lung function and respiratory muscle adaptations of endurance- and strength-trained males. *Sports*.

[53] Anastasio F., Barbuto S., Scarnecchia E. (2021). Medium-term impact of COVID-19 on pulmonary function, functional capacity and quality of life. *The European Respiratory Journal*.

[54] Mittal A., Dua A., Gupta S., Injeti E. (2021). A research update: significance of cytokine storm and diaphragm in COVID-19. *Current Research in Pharmacology and Drug Discovery*.

[55] Shi Z., de Vries H. J., Vlaar A. P. J. (2021). Diaphragm pathology in critically ill patients with COVID-19 and postmortem findings from 3 medical centers. *JAMA Internal Medicine*.

[56] Woods J. A., Hutchinson N. T., Powers S. K. (2020). The COVID-19 pandemic and physical activity. *Sports Medicine and Health Science*.

[57] Hui D. S., Wong K. T., Ko F. W. (2005). The 1-year impact of severe acute respiratory syndrome on pulmonary function, exercise capacity, and quality of life in a cohort of survivors. *Chest*.

[58] Fabre J.-B., Grelot L., Vanbiervielt W., Mazerie J., Manca R., Martin V. (2020). Managing the combined consequences of COVID-19 infection and lock-down policies on athletes: narrative review and guidelines proposal for a safe return to sport. *BMJ Open Sport & Exercise Medicine*.

[59] Buchman A. S., Boyle P. A., Leurgans S. E., Evans D. A., Bennett D. A. (2009). Pulmonary function, muscle strength, and incident mobility disability in elders. *Proceedings of the American Thoracic Society*.

[60] Huang C., Huang L., Wang Y. (2021). 6-month consequences of COVID-19 in patients discharged from hospital: a cohort study. *Lancet*.

